# The Reform of Basketball Curriculum Model for Students' Physical Development under the National Fitness Environment

**DOI:** 10.1155/2022/2869323

**Published:** 2022-07-01

**Authors:** Hui-chao Li, Shun-fa Shen

**Affiliations:** Department of Physical Education, Civil Aviation University of China, Tianjin 300300, China

## Abstract

College sports serving national fitness are a complex system. College sports are an important part of national fitness. Basketball curriculum, as a subsystem of college sports, has always been loved by college students. The reform of college basketball curriculum mode is an important way to explore the coordinated evolution of college sports subsystem. Through the methods of questionnaire, interview, and mathematical statistics, aiming at the problems existing in the planning and design of basketball curriculum objectives and contents in colleges and universities, this study puts forward that it is necessary to establish a scientific and reasonable basketball special curriculum objective system and then combine the basketball curriculum teaching theory with the basketball training teaching mode, to cultivate students' practical application ability, and adopt a variety of teaching methods to cultivate students' practical ability. Finally, the teaching mode of basketball is improved. Through an example, the application effect of the basketball curriculum model under the background of national fitness proposed in this study is tested. The results show that the basketball curriculum teaching model proposed in this study has certain feasibility and effectiveness.

## 1. Introduction

The introduction of a series of sports laws and regulations, such as the Outline of the National Fitness Program and the Sports Law, shows that the state attaches great importance to national fitness. With the promotion of national fitness, the relationship between college physical education and national fitness is becoming increasingly close and has become a key topic of research. Coordinating the relationship between college physical education and national fitness has become the foothold of implementing the national fitness plan, which has attracted extensive attention at home and abroad.

In recent years, domestic scholars have focused on the supply-side reform of college sports. As an important part of the “Healthy China” strategy, school physical education has always been a key field of the development of the party and the country [1]. Some people analyzed national fitness and college physical education reform, focusing on the direction of college physical education promoting national fitness reform [2]. Some scholars focused on improving the teaching mode of physical education in colleges and universities and enhancing students' fitness awareness in their research on ways to promote national fitness in college physical education [3]. Most of the above studies involve macro-factor analysis and lack of in-depth research at the level of physical education curricula in colleges and universities, but they provide the basis and reference for this study.

As the demand for sports is more extensive, colleges and universities should set up some sports courses to meet the needs of social development, so that college sports can meet the development of national fitness needs. In view of the above research results, through the method of questionnaire survey, interview, and mathematical statistics, this study puts forward countermeasures and suggestions for the present problems in the planning and design of the objectives and content of college basketball curricula and gives a school basketball curriculum model under national fitness context.

## 2. Analysis of the Relationship between College Physical Education and National Fitness

At present, the progress of the society has put forward higher requirements for the physical quality of people, and there are still many problems in the development of the national fitness work. To further develop the national fitness project, the supply of college physical education resources is needed. The relationship between college physical education and national fitness is getting closer and closer. College physical education resources become the running starter of national fitness, which has obvious influence and long-term benefit on national fitness. The development of national fitness is influenced by the technical guidance, information exchange, organization and management, and cultural inheritance of college sports resources. College sports resources provide human reserve and technical guidance for the development of national fitness [4].

In recent 10 years, the number of students in colleges and universities in China has been increasing year by year. In 2021, the total number of students in various forms of higher education in China is 41.83 million [5], and college students are an important force in the cause of national fitness. As the last station of physical education, scientific and reasonable college physical education can not only fully mobilize the enthusiasm of students on sports and enable them to master 1 or 2 lifelong sport projects but also cultivate students' view of sports and health and promote the achievement of teaching goals. College graduates entering the society input more sport resources for the society, create a stronger sports atmosphere, and better promote the development of the national fitness cause. Therefore, it is inevitable to require the continuous development and perfection of college physical education curriculum for the vigorous development of the national fitness movement.

According to the above analysis, the structure chart of the relationship between college physical education curriculum and national fitness is constructed, as shown in Figure 1.

College physical education can not only cultivate students to participate in sports in different ways but also promote the demand of national fitness. College physical education should pay attention to open teaching, comprehensively improve students' comprehensive quality, and establish the idea of lifelong participation in physical education.

## 3. Current Situation and Existing Problems of Curriculum Construction

### 3.1. Current Situation of Curriculum Construction

#### 3.1.1. Teaching Materials and Curriculum Construction

Ministry of Education mentioned in Give Priority to Education that talent cultivation and moral composition need to grasp the characteristics of the quality-oriented education era and focus on the construction of teaching materials and teaching reform in primary and secondary schools and colleges [6]. Some people pointed out that the setting of physical education courses in universities should consider the needs of students, start from their physical and mental characteristics, and aim at cultivating interest, stimulating interest, and forming lifelong sports habits [7]. At present, the teaching content of basketball in China mainly consists of basketball theory, basic techniques, tactics, special physical qualities, and teaching competitions. The teaching content is reasonable, but the content is not deep enough, with high repetition with primary and secondary school courses and no special basketball teaching material. Some scholars believe that quality requirement has become the new task of physical education teaching reform and is also the imperative goal of innovation in the. The creation and compilation of textbooks do not take into account the cultivation of students' personality, expertise, and interests, which is not conducive to the formation of exercise methods and habits suitable for students according to the knowledge of textbooks [8]. Through the investigation of 8 colleges and universities in Tianjin, Hebei, Beijing, and Shandong, it was found that the introduction of the subjects in college physical education textbooks is too general and that there are no detailed technical and tactical training methods, playing a very limited auxiliary role in teaching.

#### 3.1.2. Assessment Content and Scoring Standard

According to the Opinions of the General Office of the State Council on Strengthening Physical Education in Schools and Promoting All-Round Development of Students' Physical and Mental Health, physical education course assessment should highlight process management and comprehensively evaluate students' attendance, classroom performance, health knowledge, sports skills, physical health, extracurricular exercise, and participation in activities. Some people pointed out that the current physical education teaching evaluation system in China ignores the differences between individual college students due to innate genetic factors and acquired development factors and ignores the efforts of students in the learning process, which are unhealthy and unfair teaching evaluation [9, 10]. At present, the examination content of basketball skills in colleges and universities lays too much emphasis on the mastery of basketball skills but lays no emphasis on their ability to participate in basketball games, which is not conducive to the cultivation of students' sports habits. The straight and curve dribbling and three-step layup are taken as an example; the technical score accounts for 90 points, and the hit rate accounts for only 10 points. As we all know, the most important thing in basketball court is to score. In fierce confrontation, it is impossible to achieve the standard of technical movements every time. Therefore, overemphasis on “technical evaluation” is not conducive to stimulate students' enthusiasm in practice and the formation of students' sports habits.

### 3.2. Reflection on the Construction of Basketball Curriculum in China

#### 3.2.1. Basketball Course Teaching Content

School physical education curriculum is an important way to improve national physical health. The party and the state attach great importance to youth physical education and successively introduced the Outline of Teaching Guidance for Physical Education in National Colleges and Universities, the Curriculum Standard for Physical Education (Grades 1–6), and Physical Education and Health (Grades 7–12) in General Senior Middle Schools of Full-Time Compulsory Education, Decision of the CPC Central Committee and the State Council on Deepening Educational Reform and Comprehensively Promoting Quality Education, and other documents. On the whole, physical education in schools in China has built a complete teaching system and stipulated the teaching content for all ages [11]. However, when planning the teaching contents of physical education courses, the teaching departments did not make overall arrangements for the progress of primary schools, middle schools, and universities, which not only resulted in the phenomenon of repeated teaching contents but also difficult to meet the actual needs of national fitness, as shown in Table 1.

Table 1 shows that there are two problems in current basketball teaching in schools. First, there are many repetitions in basketball teaching in colleges and middle schools. Basketball skills are mostly personal skill training, and there is a lack of interactive units between students. At the university level, students should be taught the correct application of basketball skills to improve the tactics in the game. For example, the layered method can be adopted to carry out teaching competitions for students at the same level of basketball skills to increase their interest in learning [12]. Second, the means of assessment are relatively simple. The assessment contents of the middle school stage include 1-minute jump shot, three-step layup, and two-handed chest passing and that of the university stage include free throw line shooting and the straight and curve dribbling followed by a three-step layup. In terms of difficulty, the fixed-point free throw is even less than one-minute jump shot. Basketball is a team game, and only in a team can experience the fun of basketball [13]. Therefore, it is necessary to improve the assessment of students' technique and tactic application. Only by adapting to the needs of actual combat can students increase their enthusiasm for sports participation, increase their sense of achievement, make basketball have the opportunity to become an alternative project for students' sports leisure, and cultivate students' concept of lifelong sports and health.

#### 3.2.2. Student Information of Basketball Option Class

The basic basketball exercise level of students in the basketball option class determines the teaching content, teaching progress, and the application of teaching methods. The teaching content of teachers can achieve the teaching objectives only by fitting the reality of students and through classroom practice. A total of 550 questionnaires were distributed, and 541 valid questionnaires were collected from 8 colleges and universities in Tianjin, Hebei, Beijing, and Shandong. The findings are as follows.

*(1) Time for Students to Contact Basketball*. It can be seen from Figure 2 that 41.9% of the students have more than 3 years' experience of touching the ball, and 25.8% of them have 1–3 years' experience of touching the ball. It is worth noting that more than 22.7% of the students have less than 1 years' experience, and even 9.6% of the students have never touched basketball. It is very challenging for us to carry out basketball teaching and develop students' interest in basketball.

*(2) Self-Assessment of Basic Basketball Level*. As can be seen from Figure 3, students are not very satisfied with their basketball skills. Among 541 students, only 16% think their basketball skills are good or very good, while 42% think their basketball skills are poor or very poor. Therefore, we can infer that although 67.7% of students have more than one year's contact time with basketball, they just use basketball as physical education, but not as leisure sports.

*(3) Number of Times Students Participate in Basketball Every Week*. As shown in Figure 4, except for the basketball class once a week, only 31.2% of students take basketball as a physical exercise, while 68.8% of students only take part in basketball exercise once or never after class. We have carried out basketball education and teaching for more than ten years, but it remains a course for most students. They did not translate basketball sports into physical exercise and did not make basketball a priority.

*(4) Students' Motivation in Basketball Option Class*. As can be seen from the statistics in Figure 5, 94.7% of students actively choose basketball lessons, indicating that students have a strong interest in and expectation of basketball lessons.

*(5) Students' Expectation to Participate in Basketball through the Learning of Basketball Class*. It can be seen from Figure 6 that students have great expectation to participate in basketball after learning basketball courses. 81.8% of students hope to participate in basketball through learning basketball lessons. 12.9% of the students said they were not looking forward to playing basketball, but the number would continue to shrink if they were taught properly. Only 5.3% never looked forward to playing basketball.

Nearly 42% of the students think their basketball level is poor or very poor, but 67.7% of the students have more than one year of basketball contact time. 68.8% of the students have only once or never participated in basketball exercise after class, but 81.8% of the students hope to learn basketball to participate in basketball. According to the above questionnaire survey data, if we still use the traditional teaching methods and only pay attention to students' personal skills, it is not conducive to the cultivation of students' sports habits, but also completely contrary to the curriculum goal of cultivating students' lifelong health. Therefore, college basketball education should change the teaching concept and teaching means. It should be student-centered and allow students to learn from each other through teamwork. In this way, students can truly understand the environment in which basketball technology is applied, and their learning enthusiasm can be stimulated, so that students' concept of lifelong physical health can be cultivated.

According to the statistical results of the questionnaire survey of basketball elective courses, although most students have a strong interest in basketball courses, affected by traditional teaching methods, students are not satisfied with the teaching of basketball courses in China on the whole.

#### 3.2.3. Class Hour Design

The outline of “Healthy China 2030” issued in 2016 points out that it is necessary to cultivate young people's sports hobbies and basically realize that young people can master the skills of at least one sport [5]. When sports became physical education, its cultural attributes, participation obligations, content characteristics, training cycle, time and place, collective exercise, and scale of learning all changed greatly. What should have been a “long continuous specialized training process” became “a short and fragmented teaching process in physical education classroom.” This is the internal reason why “students have studied physical education for 12 years without learning anything” [14, 15]. According to the survey results in Table 1 and on-site observation, it is found that at least 50% of the students in the basketball option class have average sports skills, and nearly 40% of them have poor basketball skills. We have carried out 12 years, nearly 1260 class hours of school physical education, but most students fail to master the skills of one sport. One of the most important reasons is the unreasonable arrangement of school hours. Taking basketball teaching as an example, the whole middle school basketball teaching time is 30 class hours, and the college basketball teaching time is 34 class hours, including body test time and assessment time. This kind of unclear “comprehensive and diverse” teaching arrangement is the main reason for the ineffectiveness of the current PE curriculum. Cultivating a sport skill should be a continuous teaching process for many years. Therefore, we should appropriately adjust the current course selection methods, extend the class hours of each course, and allow students relatively enough time to deepen and improve the skill in the classroom.

#### 3.2.4. Teaching Methods

From the survey results of students' understanding of basketball course, there may also be some other factors that lead to the unsatisfactory opening of basketball elective course. For example, the modern teaching method of basketball course may be quite different from the traditional teaching mode, which makes it difficult for some students to adapt. Basketball skill is the basis of basketball. It has fixed content, but it is not limited to form. The traditional basketball course is mainly taught in the form of lectures. That is, the teacher demonstrates first, then the students carry on the imitation practice through observation, and the teacher carries on the tour guidance again. The teaching process is boring, and students' initiative in learning is not high. When learning technical movements, students only know how to do them but do not know why. Thus, when learning movement skills, they do not have a high efficiency. Although lecturing teaching can play a good effect in the early stage of students' basketball sports skill learning, it is not conducive to the in-depth understanding of basketball techniques. The traditional teaching method ignores the subjectivity of students, and the innovative teaching methods such as independent exploration, heuristics, and discussion are not used in basketball teaching. To improve students' basketball skills, we can improve the teaching methods.

## 4. Necessity of College Basketball Curriculum Mode Reform

### 4.1. Curriculum Mode Reform Should Conform to the Needs of the Times of National Fitness

Since the 18th National Congress of the Communist Party of China, the CPC Central Committee with Comrade Xi Jinping at its core attaches great importance to physical education and school physical education, emphasizes the close relationship between building a strong country through sports and the Chinese Dream, regards the construction of a healthy China as an important support for the Chinese Dream, integrates physical education and school physical education into the overall plan of realizing the “Two Centenary Goals,” and makes the nationwide fitness program a national strategy. Curriculum is the basis of education and teaching in colleges and universities, and curriculum construction is one of the important contents of school teaching reform [16]. Therefore, strengthening physical education curriculum construction is an important guarantee to effectively implement physical education teaching plan and improve teaching level and talent cultivation quality. College basketball curriculum reform should scientifically analyze and rationally understand the new situation and new challenge of the national fitness cause, and fully understand the new orientation, new direction, and new requirements of the college basketball curriculum from the strategic height and overall point of view; understand the strategic positioning of college basketball courses from the perspective of realizing the “Two Centenary Goals” and the Chinese Dream of the great rejuvenation of the Chinese nation; and promote the deepening of education and teaching reform from the height of building a healthy China and a strong country in sports.

### 4.2. Under the Background of Supply-Side Reform, Curriculum Construction Must Focus on Students' Development

On November 10, 2015, Chinese President Xi Jinping put forward the “supply-side reform” for the first time at the meeting of the Central Leading Group for Financial and Economic Affairs, pointing out that “while moderately expanding aggregate demand, we should strengthen the supply-side structural reform and improve the quality and efficiency of the supply system” [12]. On January 8, 2018, Chen Baosheng, Minister of Education, pointed out in People's Daily that the focus of strengthening school physical education work is to do a good job in teaching material construction and teaching reform in universities and primary and secondary schools [17]. These facts show the inevitability of the supply-side reform of school physical education. The essence of the supply-side reform of college education is also the fundamental embodiment of “student-centered” education. The construction of college basketball courses must consider students' basketball needs and preferences, focus on students' development, improve teaching materials and enrich teaching methods, and provide high-quality college basketball courses.

### 4.3. Both Scientific Research and Teaching Should Be Emphasized, and the Mutual Transformation between Scientific Research and Teaching Should Be Paid Attention to

As the saying goes, “As a teacher, it's important to preach and get rid of doubts.” College teachers should not only undertake the responsibility of “preach” but also cultivate students' independent personality and make them master certain ability to deal with problems by themselves [18]. This requires physical education teachers to timely track the cutting-edge information of the development of physical education, master the new methods and technologies to discover and cultivate students' physical functions, bring the ideas, methods, and progress of physical research into the field of physical education, constantly enrich the connotation of college basketball teaching, realize the feedback of scientific research on teaching, and provide a steady stream of power for college physical education. Physical education teachers in colleges and universities should not only teach students sports skills but also teach students how to exercise scientifically. This requires teachers not only to learn new knowledge but also to adhere to research and pay attention to the mutual promotion of scientific research and teaching.

### 4.4. It Is an Inevitable Trend of Discipline Construction and Development to Create Excellent Courses

In the future, the subject courses in colleges and universities must have the characteristics of first-class teachers, first-class teaching content, first-class teaching materials, first-class teaching methods, and first-class teaching management; otherwise, they will be submerged by the flood of rapidly developing knowledge [19]. The development of the Internet makes the way for students to acquire knowledge diversified, and basketball classroom is greatly challenged. The goal of basketball discipline construction is always “excellent.” It should not only teach students sports knowledge but also be “new,” that is, new teaching methods, new learning methods, and new practice methods. With the spring breeze of teaching reform and development in our school, we should develop students' physique and cultivate students' lifelong view of physical education and health.

### 4.5. The Essence of Physical Education Is to Cultivate Students' Lifelong View of Physical Health

Einstein said that the so-called education is the ability left after forgetting all the knowledge learned in school. This requires teachers not to “read” knowledge to students, but give a spiritual encouragement or inspiration that can touch or shock their hearts. What basketball class should bring to students will never be forgotten in a lifetime. Inspired by this concept, college basketball teaching should not focus on the teaching of students' basketball skills, but should encourage students to use these skills more and guide students to enjoy basketball [20]. The fundamental purpose of basketball teaching is to let students find fun and gain a sense of achievement in basketball and gradually make basketball a habit of students and accompany them for their whole life.

## 5. Methods and Measures of College Basketball Curriculum Mode Reform

### 5.1. Changing Teaching Objectives and Returning Physical Education to Its Origin

Sports skill teaching is the core content of sports teaching, and the sports curriculum system based on sports skills reflects the value of sports as an important course in school education [21]. Similarly, the learning of basketball skills is the core content of basketball teaching. However, the learning of any sports skills is ultimately for application. Basketball game is the most direct way to test basketball sports skills. The basketball game without the support of sports skills is terrible, while the learning of basketball skills without the game is boring and cannot be tested. At present, college physical education still adopts the traditional syllabus, refines the classification of physical skills, and pays attention to form and ignore results, which is contrary to the purpose of basketball sports. Therefore, *t* it is necessary to change the teaching objectives for cultivating students' basketball consciousness. We should start with cultivating students' interest in sports and the practicability of basketball skills, allow the “diversification and personalization” of basketball sports skills, and let basketball education return to the origin of physical fitness.

Around the teaching objectives of physical education courses, combined with the teaching guiding ideology of basketball special courses, the goal system of basketball special courses can be established. As shown in Figure 7, starting from the basic teaching objectives of basketball course, corresponding teaching contents are formulated for the learning objectives of different semesters and stages, to decompose the teaching objectives of basketball course layer by layer and better implement them.

### 5.2. Optimizing Teaching Content and Reducing Low-End Repetitive Content

Although we have experienced more than ten years of school physical education from primary school to university and have a complete teaching management system, there are many low-end repetitions between college basketball teaching content and middle school basketball teaching content, which wastes a lot of valuable class hours and hinders the development of students' basketball skills. Therefore, the teaching content of college basketball course should reduce the time occupied by the basic sports skills of basketball and use the saved class hours to increase the content of teaching competition, to improve the application ability of students' basketball technology. Whether basketball skills are mastered or not and whether they are good or bad must be tested in actual combat. At the same time, the fundamental purpose of learning basketball skills is sports leisure and strengthening physique. In the investigation of the factors affecting students' participation in basketball, 35.5% of the students gave up sports because of their poor basketball foundation. It can be said that many people refuse sports because they are not confident or timid, so we should provide as much teaching and competition time as possible in class. The students with little difference in skills will be divided into groups for competition, so that the students can experience the fun of teamwork and the sense of success, which will slowly guide the students to love basketball.

To train students to master various skills of basketball from the aspect of practical ability, we can combine the teaching theory of basketball course with the teaching mode of basketball training, to cultivate applied talents who love basketball. As shown in Figure 8, in the process of basketball practice teaching, students' practical application ability can be cultivated from the aspects of layered practice teaching, club practice teaching, observation training on-site teaching, basketball skill practice teaching, extracurricular training practice, bilingual practice teaching, etc.

### 5.3. Extending the Class Hours and Changing the Semester System to the Academic Year System

At present, most colleges and universities provide a variety of physical education courses for students, but students are required to complete the study of four sports within two academic years. The original intention of this policy is to “cast a wide net and catch more fish,” so that students can find the sports they are interested in and then take it as the first choice of lifelong sports. However, it ignores the students' acceptance ability. Mastering a sports skill requires long-term exercise under the guidance of teachers. It is not easy to master this motor skill in just a short period of more than 30 class hours. This contradicts the strategic requirements of “Healthy China 2030.” If we want students to master a sport, we must create opportunities for students to learn a sports skill for a long time. Therefore, it is suggested to cancel the requirement that four different courses must be selected in four semesters and to extend the class hours by changing one choice in one semester to one choice in one academic year. To take care of students' sport needs, students can be allowed to transfer out at the end of each semester according to their own needs. Adopting flexible and diverse course selection methods is not only conducive to students' finding suitable sports but also conducive to students' mastering sports skills, to lay the foundation for students' lifelong sports.

### 5.4. Being Student-Centered and Innovating Teaching Methods and Means

Basketball is an antagonistic sport in the field. The situation on the field changes rapidly. Only when students really understand the characteristics of various sports skills and flexibly use basketball skills according to the situation on the field, they can achieve better results and obtain a sense of sports achievement. In the early stage of sports skill learning, traditional lecturing method of teaching can enable students to quickly establish sports image and improve teaching efficiency, but it shows its limitations in further study of basketball sports skills. Inquiry and heuristic teaching should be properly introduced. This teaching method with students as the main body and teachers as the guide can enable students to gradually master the essentials of motor skills in the process of thinking-practice-rethinking-practice and fully mobilize students' enthusiasm in learning. The whole teaching process is easy and efficient, which is twice the result with half the effort compared with traditional teaching.

For example, in the training of basketball students' practical ability, diversified teaching methods can be adopted to combine teaching, training, observation, application, and other teaching methods. At the same time, we can adopt the means of combining inside and outside school, inside and outside class, application, and practice to cultivate students' ability, as shown in Figure 9.

In the teaching process of college basketball course, affected by the individual differences in students, if a single teaching method is adopted, it may be difficult to meet the needs of all students. Therefore, layered teaching can be adopted to meet the learning needs of students at different levels.

### 5.5. Improving the Basketball Course Evaluation System

The assessment standard is like an invisible baton, which is often the place where students spend much time practicing. Therefore, whether the assessment standard is formulated scientifically is directly related to the development of students' sports level. On the whole, there are two deficiencies in school basketball assessment methods: (1) emphasizing form and neglecting result. For example, in the three-step layup assessment, the technical score accounted for 90 points and the hit rate accounted for only 10 points. The purpose of all technical actions on the field is to serve the score. Even if the technique is good, your efforts will be in vain if you do not score in the final shot. It can be said that the hit rate is an important index to test students' psychology and physiology. Therefore, it is suggested to increase the score proportion of hit rate and reduce the score proportion of technical action. (2) The assessment content is not perfect. From primary school to university, the content of basketball assessment has hardly changed. In particular, the setting of fixed-point shooting makes students with poor basketball skills spend a lot of time practicing shooting in each class, which is very unfavorable for improving basketball skills. Basketball is a combination of dribbling and shooting, and the key to improve sports skills is movement. In the actual game, the opponent will not give you time to stand in place and shoot. Therefore, it is suggested to reduce the proportion of technical evaluation scores, increase process evaluation scores, and cooperate with the application of case teaching. This can not only mobilize students' enthusiasm for learning but also greatly promote students' mastery of basketball skills.

In the process of basketball practice teaching, on the basis of mastering the basic situation of students, instructors can divide students into different levels to make students study in a more suitable environment [22]. Students at each level can carry out teaching according to different teaching objectives and requirements. Students at different levels help each other, learn from each other and improve together, and then evaluate according to the corresponding standards in the assessment and evaluation, as shown in Figure 10.

## 6. Implementation Effect and Evaluation of Teaching Mode

To test the feasibility and effectiveness of the basketball course model proposed in this study in teaching application, the class of basketball optional course in a university is selected as the object for experimental teaching. According to the existing teaching plan and without affecting the class groups, the students were randomly tested, and the classes with no significant difference between the two groups were used as the experimental group and the control group, respectively. Suppose class 1 is the control group and class 2 is the experimental group, with 30 people in each class. The control group used the traditional teaching mode, and the experimental group used the modern basketball teaching mode. Through the teaching experiment, under the condition that the examination method, content, and standard are the same, the theoretical and practical effects of the two classes of students are examined at the same time.

### 6.1. Comparison of Teaching Effect Test

From the comparison of theoretical examination results, it is found that the two groups of students have a better grasp of the theoretical level. Among them, the average score of the control group was 82.4, while the average score of the experimental group was 85.7. After testing, there was no significant difference between the two groups. From the comparison of physical fitness examination results, it is found that although different teaching modes have a certain impact on physical fitness, there is no significant difference between the two groups. However, from the comparison results of the examination results of basketball skills and application ability, the average scores of the students in the experimental group are 93.5 and 89.4, respectively, and their average scores are higher than those in the control group. After testing, there are significant differences between the two groups. It can be seen that the teaching mode of basketball course proposed in this study mainly focuses on the learning of basketball skills, and the teaching content is also optimized, so that students can participate in every link of teaching. Therefore, when students' basketball technical ability is improved to a certain extent, they will soon be recognized by the team. The self-confidence obtained from the team also promotes students' enthusiasm in training, and the teaching effect will soon appear. The teaching effect comparison results of the two groups of students are shown in Table 2.

### 6.2. Students' Evaluation and Comparison of Basketball Teaching Mode

To obtain the students' evaluation results of the basketball course teaching mode proposed in this study, the experiment uses the form of questionnaire to investigate the impact of the basketball course teaching mode on students' sports and mainly evaluates the performance of students from three aspects: emotional change, sports motivation, and collective self-esteem. Each evaluation index is expressed by mean and standard deviation, and the later data are processed by statistical software. From the final results, the evaluation results of students in the experimental group in learning well-being, learning interest, and collective self-esteem are significantly higher than those in the control group, as shown in Table 3. It can be seen that the basketball curriculum model proposed in this study can stimulate students' internal motivation and fully display students' personality development, to meet students' sports needs and strengthen the cohesion of the team to a certain extent.

According to the questionnaire survey results of each group on the evaluation of basketball course teaching mode, the evaluation of students in the experimental group on teaching organization methods, learning interest, and other indicators is above the good level, as shown in Figure 11. Therefore, students are satisfied with the basketball teaching model proposed in this study.

## 7. Conclusion

As a popular sport, basketball is not restricted by age and gender. It can not only enhance physical fitness and promote health but also enrich people's amateur cultural life, being deeply loved by the masses of the people. As the last stop of school education, colleges and universities are important incubators of sports population, and the development of basketball courses affects the development of national fitness plan to a great extent. In view of the problems existing in the teaching of basketball course in colleges and universities, this study puts forward some ways to cultivate students' practical ability by perfecting the goal of basketball special course, improving the teaching mode of basketball course, and comprehensively using a variety of teaching methods. Finally, an example is given to test the application effect of the basketball curriculum model under the background of national fitness. The results show that the basketball curriculum teaching model proposed in this study is better than the traditional model. Under the background that national fitness has been promoted as a national strategy, improving and developing the basketball curriculum mode in colleges and universities are conducive to cultivating students' lifelong view of sports health, which is of great significance to the realization of “Healthy China 2030.”

## Figures and Tables

**Figure 1:** Relationship between physical education curriculum and national fitness system in colleges and universities.

**Figure 2:** Statistics of students' contact time with basketball.

**Figure 3:** Self-assessment of basic basketball level.

**Figure 4:** Statistics of times students participate in basketball every week.

**Figure 5:** Statistical results of course selection motivation.

**Figure 6:** Statistics of expectations for participating in basketball through learning basketball lessons.

**Figure 7:** Schematic diagram of teaching goal design system of basketball course.

**Figure 8:** Schematic diagram of key points of basketball practical teaching.

**Figure 9:** Decomposition diagram of basketball practice teaching method.

**Figure 10:** Decomposition diagram of hierarchical teaching evaluation system.

**Figure 11:** Comparison of the proportion of students in the two groups with good teaching evaluation.

**Table 1:** Comparison of basketball teaching content between colleges and middle schools.

Content school	Middle school basketball syllabus	College basketball syllabus
Dribble	(1) Straight and curve dribbling	(1) Straight and curve dribbling
	(2) In situ cross-step breakthrough	(2) High and low dribbling
	(3) In situ ipsilateral breakthrough	(3) Swerving dribble
Passing and catching	(1) Two-handed chest passing	(1) Two-handed chest passing
	(2) Two-handed overhead passing	(2) Two-handed overhead passing and catching
	(3) One-handed shoulder passing	(3) One-handed shoulder passing
	(4) One-handed rebound passing	(4) One- and two-handed rebound passing and catching
Footwork	(1) Turn: front turn, back turn	(1) Running: varied direction running, sideways running, backward running, varied pace running
	(2) Emergency stop: jump emergency stop, step emergency stop	(2) Jump: jump on both feet or on one foot
	(3) Slide step: side slide step, back and forth slide	(3) Emergency stop: step, jump stop
		(4) Turn: front turn, back turn
		(5) Slide step: side slide step
Shooting	(1) One-handed shoulder shot	(1) One-handed shoulder shot in situ
	(2) Layups on the move	(2) Two-handed chest shot in situ
	(3) Jump shot	(3) One-handed running underhand shot
Tactics	(1) Defensive tactics: man-to-man defense	(1) Introduction to fast break (attack and defense): two on one, three on two
		(2) Introduction to joint defense (attack and defense): two-on-two formation
		(3) Introduction to tactics: man to man in half-court
Special physical quality	No	(1) Speed: 30–50 m acceleration
		(2) Strength: sit-ups, push-ups, supine leg lifts, etc.
		(3) Endurance: middle-distance race of various distances
		(4) Flexibility and coordination exercises
Examine	(1) Minute jump shot	(1) A straight and curve dribbling followed by a three-step layup
	(2) Three-step layup	(2) Shot
	(3) Two-handed chest passing	
Credit hour	30	34

**Table 2:** Comparison results of teaching implementation effects between the two groups.

Item	Teaching theory test	Physical fitness test	Practical skill test	Application ability test
Control group	82.4	84.8	86.3	83.6
Experimental group	85.7	86.2	93.5	89.4
*P*	>0.05	>0.05	<0.05	<0.05

**Table 3:** Comparison of students' psychological evaluation results after practical teaching.

Item	Emotional change	Sports motivation	Collective self-esteem
Control group	18.35 ± 2.56	37.58 ± 4.27	83.52 ± 8.16
Experimental group	22.27 ± 2.83	41.35 ± 4.63	89.26 ± 8.47
*T*	2.164	2.263	3.472
*P*	<0.05	<0.05	<0.05

## Data Availability

The labeled data set used to support the findings of this study is available from the corresponding author upon request.
